The article "Work Emotion Intervention and Guidance Training Method for Enterprise Employees Based on Virtual Reality" was retracted in 2024. Reasons: signs of a paper mill; suspected computer-generated content; unreliable results or conclusions; lack of ethics approval or compliance.

# Work Emotion Intervention and Guidance Training Method for Enterprise Employees Based on Virtual Reality

**DOI:** 10.1155/2022/3909734

**Published:** 2022-06-06

**Authors:** Lixun Zhu

**Affiliations:** University of Shanghai for Science and Technology, Shanghai 200093, China

## Abstract

**Objective:**

Improper management of employees' emotions has a great impact on work status and work efficiency, and emotional management has increasingly become a very important part of corporate human resource management. How to adjust the various emotions of employees, so that employees can work in a fuller and more passionate attitude, is a problem that enterprise managers need to consider. From the perspective of employees themselves, a good mood will also bring happiness and satisfaction to life and work. Only in this way can the company and the employees be satisfied with each other and continue to maintain the good development momentum of the company.

**Method:**

This paper proposes a new method of using virtual reality scenes to induce human emotions. Based on computer science and psychological cognitive science, a scene library of “virtual reality emotion induction system” is constructed. Emotion induction based on virtual reality scenes has better interactivity and generalization, as well as stronger immersion and user operability. Its emotional arousal is high, the data is reliable, and the interference of environmental factors in the induction process is weakened, and relatively objective emotional data can be obtained. The factors affecting the emotional management of the enterprise are investigated by means of a questionnaire survey, statistics and problems are found, and the objective problems existing in the emotional management work of the company are determined. According to the analysis, the problems are summarized, and it is believed that the company still has certain room for improvement and improvement potential in terms of corporate culture construction, emotional counseling system construction, and human resource career planning. In the research of this paper, through the combination of theory and practice, the enterprise's emotional management work has been comprehensively analyzed, and the practical problems existing in its emotional management work have been found through questionnaires. *Results/Discussion.* In the field of enterprise human resource management, emotion management is always an eternal topic worthy of our attention. But unfortunately, emotional management has not been given enough attention by managers. Most companies often think that emotions are their own business. Employees should self-regulate, control, and tolerate themselves. They should not bring personal emotions to work and even think that emotional work is unprofessional. This kind of misunderstanding has led to the fact that emotional management has not received due attention and affirmation in many enterprises.

## 1. Introduction

In the context of a globalized economy, with the acceleration of the iteration speed of technical tools, such as information tools and means of transportation, the quality of people's work and life is constantly improving, and the rhythm of work and life is also accelerating [1]. “Fast” has become the core feature of modern society in the 21st century. The complex and changeable social environment and tight working hours have brought greater work pressure to employees [2]. Work stress has become one of the problems faced by workers all over the world, and it has become a normalized and full-staffing problem.

In recent years, the employees of the company have been suffering from sudden diseases, such as karoshi and sudden death, which seriously endangered the safety of employees [3]. In addition, employees have many mental problems due to greater work pressure, such as depression, emotional exhaustion, mental exhaustion, and excessive anxiety. The workplace stress report shows that 60% of people experience anxiety or even depression because of excessive stress [4]. Excessive work pressure not only brings serious health and economic losses to individuals but also has a huge negative impact on the entire society. Work stress is no longer a personal issue but has gradually become an important issue of common concern for companies, society, and the world [5].

At present, most employees in enterprises are troubled by negative emotions, but they lack understanding of emotional management and its importance and even have less knowledge about how to improve their emotional management ability [6, 7]. Therefore, how to use the professional methods of corporate social work to better serve the emotional management of employees is a profound proposition that we urgently need to discuss.

In the process of research and intervention, it enriches and expands the theoretical basis of corporate social work and employee emotional management and tries to solve practical problems encountered by employees in the process of emotional management by combining rational emotional therapy mode and group work [8]. This itself is also an extension and expansion of the theory of corporate social work and employee emotion management, which will provide a corresponding theoretical basis for the development of such research work in the future, which is of great significance.

There are many ways to induce emotions, including visually induced text, images, and auditory induced sounds [9]. At present, the most widely used induction systems in the world are the International Affective Picture System (IAPS) and the International Affective Digitized Sound System (IADS). However, simple image or audio material is relatively low in emotion-induced ecoefficiency and poor in immersion. And in the process of inducing directional emotion, traditional induction methods are easily affected by environmental factors and must be strictly controlled in a standard environmental space [10–12].

Based on computer science and psychological cognitive science, this paper designs and establishes a “virtual reality emotion induction system.” By extracting multimodal emotion features from a low-dimensional emotion-inducing system that meets psychological standards, we design and produce emotion-inducing VR scenes and further expand to version 2.0. The object of this study, as an advanced enterprise in the industry, recognized the importance of emotional management earlier but encountered many problems in the process of emotional management, and the effect was not good.

This paper makes a systematic analysis of the emotional management problems that have been carried out, finds problems, and proposes solutions. This research not only provides necessary theoretical support for enterprises to further standardize and optimize emotional management but also provides some new ideas for enterprises to better carry out emotional management of knowledge workers. The research results of this paper can not only provide certain support for the improvement of the work efficiency of enterprise employees but also have certain reference for the formulation of emotional management solutions for designers in other industries.

## 2. Methods

### 2.1. System Framework and Design

#### 2.1.1. Overall System Architecture

The 1.0 version of the virtual reality emotion induction system includes 8 self-made virtual reality scenes, which are used to induce five basic emotions of “joy, disgust, sadness, fear, and calm,” and the duration of each scene is 80 s. Further, in AVRS 2.0 version, 16 emotional VR scenes are expanded to form 24 emotional scenes, including 8 positive emotional scenes, 8 negative emotional scenes, and 8 neutral emotional scenes.

Based on the self-assessment model emotion scoring system, the emotion evaluation of each scene is carried out, and the emotional quantification results of each scene in line with psychological standards are obtained.

This paper adopts the classic three-dimensional model of emotion (pleasure, arousal, and dominance), as the evaluation content, and selects the two most important emotional dimensions, pleasure and arousal, as the evaluation criteria. In the self-made VR scene library, in order to evenly distribute VR scenes in the emotional space, two emotional dimensions of pleasure and arousal were selected to divide the emotional space into four quadrants. Among the three emotional attributes, positive, neutral, and negative, five basic emotions (joy, fear, disgust, sadness, and calm) are selected as the initial position for scene production. And based on this, the scene is expanded to ensure that the VR produced can induce a wide range of emotions.

Based on the SAM emotion scoring system, each VR scene in the system is evaluated and corrected. We compare the evaluation results with the target emotional coordinates. If there is no significant difference, the scene is considered to be standardized. If consistency cannot be achieved, we adjust the VR scene according to the deviation until the evaluation results meet the standard.

The emotion types and three-dimensional quantitative labels obtained by SAM evaluation together with VR scenes constitute a virtual reality emotion system. Since virtual reality is highly immersive, the system can trigger emotions more effectively and accurately in the process of emotion induction, shield external interference to a certain extent, and obtain relatively objective emotional data, so as to solve the problem of immersion in existing induced materials [13, 14].

#### 2.1.2. Create the Overall Design of the Scheme

In order to ensure the scientificity and effectiveness of the “virtual reality emotion induction system,” the system was created and designed based on the emotional characteristics in the standardized low-dimensional emotional system.

Firstly, emotional features are extracted from the multidimensional emotional induction database. By screening the existing emotional design materials, a series of characteristic elements related to emotions are extracted, including color, theme, and sound, to provide a basis for the design of the virtual reality emotional scene library. Then, according to the extracted feature elements associated with emotions, based on the psychological emotion induction paradigm and VR production technology, a series of virtual reality scenes that can induce different emotions are designed and produced through Unreal Engine. Finally, through the strict psychological SAM scale evaluation, the emotional labels of each scene are obtained, and it is verified whether it reaches the standard of emotional induction system in the field of psychology, and a standardized VR emotional induction material library is formed.

After the system is established, four virtual reality scenes are put into LCD and virtual reality equipment, respectively, and the emotional arousal level is tested by heart rate and SAM scale to further test whether virtual reality scenes have advantages in emotional arousal.

### 2.2. System Creation Process

#### 2.2.1. Select the Target Emotion

The pleasure-arousal emotional space is divided into four parts: high − pleasure and high − arousal valence = 5 ~ 9, arousal = 5 ~ 9; high − pleasure and low − arousal valence = 5 ~ 9, arousal = 1 ~ 5; low − pleasure and high − arousal valence = 1 ~ 5, arousal = 5 ~ 9; and low − pleasantness and low − arousal valence = 1 ~ 5, arousal = 1 ~ 5. In the low-pleasure and low-arousal space, two emotions, sadness and disgust, with their own characteristics, were selected, and the target emotions were composed of “joy,” “disgust,” “sorrow,” “fear,” and “calm.” The target emotion positioning is shown in Table 1.

#### 2.2.2. Emotion Feature Extraction

After determining the target emotion, based on the mean value of arousal and dominance, the audio (IADS and CADS), video (CAVS), and image (IAPS and CAPS) materials are clustered according to the target emotion and screened.

For each emotion type, we select batches of low-dimensional materials (images, audios, and videos) that are consistent with their emotional coordinate regions and extract a series of emotion-related feature elements. The emotional features of each dimension are shown in Table 2.

Vision is the most important part of emotion induction, and color is the most important visual emotional element [15]. This paper generates various emotional color palettes by extracting the theme colors of the entire visual picture and provides a complete color palette guide for the establishment of VR emotion induction system. Based on the image library of the existing emotion tags, the feature extraction of the theme color is carried out, so as to determine the color features used to induce each target emotion.

The tree is constructed by traversing the input pixel color information. Each color data is inserted into the tree, and after insertion, it is judged whether the number of child nodes overflows.

In case of overflow, one of the nodes is merged. Data from all child nodes that have it as a parent is merged into this node.

Because sibling nodes with the same parent have the same high-order value, they are concentrated in a relatively similar color range. Therefore, when merging colors, we start from the bottom layer, select a suitable merged node, merge its leaf nodes, and then delete the leaf nodes. Thus, a deepest node is completed, which is also the node that has the least impact on the theme color.

The principle of the octree algorithm determines its problem in theme color extraction, that is, since the number of leaf nodes to be cut each time cannot be controlled, it completely depends on the number of child nodes under its parent node [16, 17]. That is, at most seven nodes will be removed at a time, but only one will be added. As a result, the final number of theme colors cannot be strictly controlled. In order to get enough theme colors, the number of colors in the algorithm is generally increased by force, and the color with the most pixels is selected [12]. However, in the application scenario of this topic, what this paper needs is not a certain number of colors, but a color block that really plays a big role in emotional images [18, 19]. The algorithmic disadvantage of octree becomes an advantage instead, which avoids the small proportion.

The subject color extraction of the image based on the octree produces a color data without a fixed palette. It has a strong advantage in the fidelity of the original image and has strong flexibility. Images can even be fidelity and restoration in the cache. We extract the theme color of each image with emotional labels to get the theme color ranking of a single image. According to the weight of each hue extracted from a single image, the theme color block is obtained. For the audio in the scene emotion design material, the audio in the IADS, an internationally authoritative emotional audio database in the field of psychology, and the audio in the CADS audio database, which is more suitable for eliciting Chinese emotions, are divided into five categories according to five target emotions based on their emotional tags. We extract the theme, melody, sound, and rhythm features of the audio, while expanding the theme audio resources set by the complex plot.

For the video in the scene emotion design material, we extract the plot and extend the design. At the same time, we set the lens switching rate and camera moving path and moving speed and mark the phase and moving speed of each model object.

According to psychological research, the five types of emotions can have obvious arousal signs after 46 s. At the same time, considering the emotional weakness caused by long-term induction and the technical limitations of VR technology, this paper uses the duration of each VR emotion induction scene. At the same time, the scene light source type and light change characteristics are extracted.

#### 2.2.3. Create VR Scene

According to the extracted image and theme color wheel, the panoramic design of VR scene is carried out. We set the light source type and route transformation at the same time. The goal of this step is to design the visual landscape based on the emotional characteristics of the scene guidance guide. The background environment image related to joy in each standard emotion library is extracted as the foreground image feature of the forest. Set the light source type to point light source and the light source variable to natural light transformation.

According to the extracted audio features, the joy audio related to the natural landscape in the standard audio emotion library is selected, and other related audios that meet its audio characteristics are expanded. According to the plot feature extraction of the standard video emotion library, the landscape transformation design of the scene and the plot story setting are carried out. First, the scene terrain transformation is performed. Then, this paper designs the network skeleton object and renders the sticker, sets the properties of the network skeleton object as the object control, determines its phase coordinates, size, and animation effect, and triggers conditions, movement path, and movement rate.

We add the scene light source, set the light source type, set the light source path and change function based on the blueprint, add the camera, specify the movement path of the user master character, bind the camera to the user master character, and set the movement rate and acceleration. This article adds audio and trigger controls to the model that can emit sound and sets the audio loop frequency and duration.

Finally, we add full-scene background sound effects, set up touch modules, and conduct effect tests, including dizziness tests and scene content tests.

### 2.3. The Application of the Questionnaire Survey Method

#### 2.3.1. The Purpose and Object of the Investigation

In order to better understand the basic situation of the enterprise's emotional management work, and to understand the emotional status of the employees in the hospital, the factors that affect their emotions, and the actual ability of emotions to affect their work, we choose the questionnaire survey method to collect specific data.

This questionnaire is mainly aimed at the front-line designers of the enterprise, and the coverage is good. Because they have worked in the human resource management department of the enterprise for nearly six years, they have a stable and good interpersonal relationship. With the support and help of the enterprise leaders, all colleagues have also given full support to this survey.

#### 2.3.2. Investigation Method and Content

In the data collection process of this questionnaire, quantitative investigation and analysis method is used intensively, and predesigned questions are presented to the respondents in the form of questionnaires, so as to obtain their subjective feeling data. At the same time, in the design, in order to ensure that employees can express their own thoughts without worries, an anonymous survey method is adopted. The questionnaire does not involve any employee privacy content, so as to maximize the display of employees' true thoughts.

### 2.4. Questionnaire Design, Distribution, and Recovery

#### 2.4.1. Questionnaire Design

The questionnaire design refers to the mature scale, and the first part is a survey to test the demographic characteristics of employees. From the basic level, we can understand the ratio of men and women, age structure, working years, and cultural quality level in the company, verify the characteristics of the company's personnel, and provide a basis for the investigation of emotional management factors.

The second part is the investigation of emotional management factors, which is the focus of this questionnaire. In the theoretical review part, we have mastered the characteristics and functions of emotions, what are the main motivational factors that affect emotions, and the relationship between emotion management and corporate performance, especially the theory of emotion management incentives in detail. According to the comprehensive incentive theory, the environmental factor is the physical living environment factor as the first dimension; the construction of psychological environmental factors such as fairness, satisfaction, and awareness is the second dimension as the category of corporate culture. The third dimension is the category of human resource management and development. In the first dimension of physical living environment factors, we have selected three criteria: office environment, hardware facilities, and corporate industry status.

The working physical environment includes a series of factors such as the light, humidity, and noise of the office, the size of the place, and the applicability of work tools and equipment. In addition, the soft working environment, i.e., industry characteristics, corporate industry status, and other factors also has an impact on employee emotional factors.

The second dimension is the category of corporate culture. Cultural ceremonies can use the frequency of cultural and recreational activities to reflect the lively ceremonies, such as various recognitions and gatherings of enterprises, and interpersonal relationships are the communication channels that most directly reflect the cultural network.

In the end, we chose the following five criteria: corporate cultural atmosphere, corporate values, interpersonal relationships, management system, and frequency of recreational activities.

#### 2.4.2. Questionnaire Distribution and Recovery

In order to improve the efficiency of this questionnaire and reduce the difficulty of operation, this questionnaire was distributed on the WeChat platform, and the design process fully considered the industry characteristics of the design industry and the general characteristics of knowledge workers. It is hoped that this questionnaire can provide detailed and effective first-hand data for the smooth development of this research, so as to provide sufficient data support for a better understanding and diagnosis of the current situation of emotional management in enterprises.

The recovery rate for this survey was 100%. Excluding the questionnaires with obvious errors and clearly not meeting the requirements, the finally obtained questionnaires have an effective rate of about 96%. This questionnaire is only aimed at the company's grass-root employees, and the sample size is also sufficiently large. During the investigation process, the main object is the employees in the front-line design positions, who have a good ability to respond to the management situation of the company.

### 2.5. Construction of Enterprise Employee Emotional Management System

#### 2.5.1. Cultivation Mechanism

In practice, the specific measures for the emotional management and regulation of enterprise employees should be combined and integrated with the system, process, and cultural construction of the enterprise, so that the entire employee emotional management system can truly be deeply rooted in the hearts of the people. In addition, the establishment of emotional incentive system can stimulate the vitality of enterprises. The employee's emotional performance is summarized into the performance evaluation, and there must be punishment and reward, which can stimulate the internal motivation of employees. At the same time, improving the welfare of employees and providing development opportunities can effectively supplement the physical and mental resources of employees and stimulate their enthusiasm and enthusiasm for work. The emotional management system constructed in this paper is shown in Figure 1. Enterprises must create more favorable emotional management according to the corporate environment.

At the same time, they must establish correct emotions and emotional management concepts, so as to ensure that company employees face up to the essence and importance of emotional management, which is conducive to creating a better culture atmosphere, thereby enhancing the cohesion of the team and even the entire company. In addition, mutual help and encouragement among employees can also improve employee work performance to a certain extent.

Finally, the system must be optimized from all aspects, so that the cultivated emotional atmosphere can be better developed.

#### 2.5.2. Intervention Mechanism

The company's human intervention in the employee's emotional management system is an active adjustment mechanism. Enterprises should mobilize the initiative of emotional management, inspect the artificial system intervention, and then solve emotional problems in real time, which can more effectively prevent the breeding of negative emotions and at the same time is conducive to reasonable and effective management of employees' emotions. Strengthening the awareness of emotions among corporate staff is the most important measure to prevent emotional problems. Enterprises should organize all activities that can improve the “emotional cognition level,” such as training and seminars, and establish various learning platforms or interest groups. Helping corporate members to strengthen the ability of personal emotional management can also strengthen the ability of other aspects of employees. Human intervention is the main measure of the intervention mechanism. The superior leaders should always pay attention to the emotional changes of employees and can take the initiative to prevent and help employees to manage and regulate their emotions. A unique corporate culture has been established based on the working emotions of the employees, and the emotional IQ of the employees has been improved. On this basis, the company's corporate culture construction will be improved from a strategic perspective, and top-down attention will be paid to it.

At the same time, through the improvement of various management systems, such as distribution, the sense of ownership of employees is enhanced, so that all employees feel that they are equal members of the company, and they will not be discriminated and treated unfairly, eliminating frustration and imbalance.

It is necessary to intensify efforts to build a corporate spiritual culture, so that employees can support colleagues and care about customers to establish a harmonious employee relationship, help employees handle the relationship in life, and create a family-style emotional atmosphere of mutual respect, mutual understanding, and harmonious progress.

#### 2.5.3. Grooming Mechanism

It is an important part of the whole emotional management system to establish an emotional management mechanism dominated by the emotional problem relief mechanism. Enterprises need to understand the nature of emotions, focus on “dredging,” establish a systematic and comprehensive emotional dredging platform, which can help people who have emotional fluctuations or negative emotions due to various reasons to release their emotions appropriately, and further strengthen the platform. Communication and counseling between employees stabilize the emotional atmosphere of the company's work. Apart from formal system and cultural construction, managers should update their concepts, pay attention to the guidance of employees' emotions, and encourage various spontaneous and informal communication channels.

## 3. Results

### 3.1. Analysis of the Survey Results of the Statistical Characteristics of Enterprise Employees

According to the questionnaires received, the results of the survey on the basic information of employees are shown in Table 3.

From the male-to-female ratio of designers, it is not difficult to see that there are more males and fewer females in enterprises, with a ratio of about 3 : 1. This phenomenon is due to the characteristics of the industry. The design industry has a lot of work pressure, working overtime, and staying up late. When encountering urgent tasks or large-scale design operations, the operation team often works overtime overnight for several consecutive nights. In addition, designers need to go out to the construction site frequently, and men have an advantage over women in terms of physical strength. Women generally work until around the age of 30, especially after starting a family and having children, and it is difficult to do high-intensity and stressful work. After pregnancy, some female designers usually do not choose to take maternity leave but directly submit resignation applications, because they do not want to continue working hard and prefer to rest and recuperate. In addition, another reason for the ratio of male to female in the company is that the company artificially controls the recruitment process to 3 : 1.

During this investigation, it was found that most of the company's main designers were post-80s employees. From the analysis of personnel structure, the post-70s and post-80s generations of the company occupy an absolute position as the backbone linking the past and the next. As experienced experts, the post-60s lead and represent the professional status of the enterprise, while the new generation post-90s absorb less, and in the long run, the follow-up motivation of personnel needs to be increased. Of course, for emotional management, the post-70s and post-80s generation are more mature and stable in the workplace, and emotional management is easier to operate and control than the new generation.

According to the data obtained in this survey, it can be found that the employees of the company generally have a relatively long working experience, and a considerable number of people have worked here shortly after the company was established. At the current stage of the enterprise, the working years of employees are generally longer, and there are certain advantages in work experience. However, long-term work can easily lead to slack in emotional management, which is also very common.

### 3.2. Analysis of the Survey Results of Emotional Management Factors

#### 3.2.1. Corporate Culture

The scope of corporate culture is very broad. Generally speaking, it includes a series of elements such as a company's values, codes of conduct, historical traditions, ethics, corporate systems, and corporate products. It penetrates and is reflected in all aspects of the operation of the enterprise.

In this section, we calculate the total score for each option for an intuitive horizontal comparison.  Figure 2 shows the number of people with different ratings of cultural atmosphere, which shows that there is still room for improvement in corporate cultural atmosphere.

In the issue of interpersonal relationships, it is very different from cultural atmosphere and cultural values. In enterprises, most employees are more aware of interpersonal relationships. This is also related to the characteristics of the designer's own work. Because the work pressure is high, the work is relatively busy, the employees spend a long time on the work content itself, and the interpersonal communication is relatively simple and direct. Although as a knowledge worker, there are deeper requirements for interpersonal communication, the busyness of work itself restricts the complexity of interpersonal communication in the company. In addition, the system of corporate entertainment activities should also play a good role to some extent, making the interpersonal relationship between employees smoother and more active, especially within the department, and the relationship is more harmonious.  Figure 3 shows the number of people with different ratings of interpersonal relationships.

#### 3.2.2. Human Resource Management and Development

As the most important resource of a modern enterprise, people have a significant impact on the enterprise. With the development of modern enterprises, the management and development of human resources has been paid more and more attention by scholars, experts, and entrepreneurs [3, 8, 11]. According to the design of the questionnaire, combined with the actual situation of the enterprise, we set the following three questions. The question setting and evaluation of human resource management and development are shown in Table 4.

In the dimension of performance incentive, employee evaluation tends to be positive. Due to the need for listing, the company has adopted a higher level in the industry from the very beginning in terms of salary design. The performance appraisal mechanism has been continuously revised and improved for six years since the first edition of the performance appraisal specification in 2018 and has achieved good results in quantifying the work results of designers and evaluating the design level. There is a special drawing review department in the courtyard, which specially grades and evaluates each drawing produced by the designer and tracks the quantity and quality of work in real time. Therefore, we can clearly observe this achievement in the network diagram.

Employees are dissatisfied with training on emotion management. In terms of human resource management, there is no emphasis on training and development of employee emotional management. Since the implementation of emotional management, the company has only conducted two training sessions. There is neither targeted training according to the situation of employees nor leaders who have a deep understanding of the situation of the company to conduct emotional management training.

#### 3.2.3. Publicity and Guidance

Setting this dimension can more intuitively see the employees' understanding and cognition of emotional management and clearly show the employees' evaluation of the company's emotional management results. The problem setting and evaluation of publicity and grooming are shown in Table 5.

The purpose of the question “Do you understand emotional management” is to better understand the cognitive situation of emotional management in the designer community, and it also shows the ability of employees' emotional management from the side. Employees do not fully understand emotion management. Although the company has carried out emotional management, employees are still not well absorbed and accepted. The ability to manage emotions without understanding natural emotion management has not been developed and exercised relatively professionally and systematically. The objective existence of the above situation proves that most of the employees in the current stage have insufficient basic knowledge of emotional management. This requires managers to further publicize the importance and necessity of emotional management in the future.

Enterprises have not done a good job of training and development for emotional management issues, have not done a good job of publicity, and have not actively organized emotional management activities. Even though the management has noticed the importance of emotional management and implemented emotional management methods, it has not been well passed on to employees. This is a problem that managers should pay attention to.

### 3.3. Analysis of the Results of Auxiliary Problems

#### 3.3.1. Happiness at Work

The weight of work happiness is shown in Figure 4. Through a simple analysis of the survey data, we can find that 34.13% of the employees of the company think that they are not happy at present, while 50% of the employees think that they are unhappy. This is a very dangerous data. The objective existence of the above situation proves that at the current stage, the employees of the company as a whole have not been able to feel happy at work.

In response to the above situation, on the one hand, the managers of the enterprise should pay due attention and attention to the lives of employees, and on the other hand, they should also make targeted adjustments to the existing management methods to help the positive transformation of employees' emotions. In addition, 11.11% of employees said that they can gain happiness from their work. These employees are undoubtedly a very valuable asset for enterprises and should be more actively guided. Another 4.76% of employees said that they did not know whether they were happy at work, which may have something to do with the differences in employees' personal perceptions.

#### 3.3.2. Frequency of Bad Emotions

Objectively speaking, human emotions often have cyclical characteristics, and everyone will have bad emotions, but different people have certain differences in the frequency of bad emotions. In order to better understand the current situation of emotional management at the current stage, we also included this question into the questionnaire, which can also reflect the basic level of the emotional management work of the hospital at the current stage.

In this question, 70% of the interviewed employees said that they occasionally have bad emotions. This data shows that employees' emotions are in a controllable state most of the time, and it also proves that companies have achieved good results in emotional management. At the same time, 24% of employees said that they often have bad emotions, and these people are obviously the ones who need to focus on the development of emotional management in the future. We must realize that negative emotions are contagious at work. If we cannot get effective control and targeted management, it will definitely bring serious negative impact on the overall operation of the company. Another 3% of employees said that they rarely have bad emotions, and these employees are undoubtedly an important force to enhance the brand image for the company.

In addition, the frequency of adverse emotions before and after the emotional intervention of virtual reality technology is shown in Figure 5. It can be seen that after the emotional intervention of virtual reality technology, the frequency of bad emotions has been significantly reduced.

## 4. Discussion

### 4.1. Self-Avatars in Virtual Reality Scenarios

Head-mounted display virtual reality systems revolve around the user's vision. A side effect of this is that users cannot see their own bodies. Thus, such systems typically include a virtual representation of the body depicted from the first-person perspective of the user's eyes [20]. Such self-avatars have obvious immediate benefits: they can give obvious clues about the user's position in the virtual world and the user's current body posture.

When embodied in an avatar, in some ways the user sees the avatar as their entity. The use of self-avatars has now been extensively studied in virtual reality, in part because virtual reality has proven to be a flexible medium in which the perceptual experience of experimental participants can be controlled. This field grew out of a pioneering demonstration of the rubber hand illusion, in which participants believed that the rubber hand was part of their body. Variations of this demonstration have taken place in virtual reality, showing that virtual limbs can be experienced in some way as part of the body or as a representation of the body.

The use of self-avatars in immersive virtual reality systems has been shown to have significant effects on spatial presence, interaction, and perception [21, 22]. Although the utility of self-avatars has been shown for specific interaction tasks, the presence of self-avatars contributes to the general performance of tasks in virtual worlds. In particular, self-avatars can help perform tasks that can be accomplished through reasoning and imagining rather than manipulation [23]. Active interaction and cognitive theories allow humans to load mental tasks into the physical world.

So making sketches on paper or manipulating pieces in a game can help in making decisions [24]. Additionally, gestures such as pantomime can act as proxies for actual manipulation or movement. If these theories are correct, the lack of self-incarnation may hinder this process of loading mental tasks so that task performance requires more cognitive load [25]. The researchers demonstrated that self-avatars can help participants' cognitive processes while being immersed in a virtual reality system [4, 12, 26]. The results further demonstrate the importance of proper self-avatar representation in immersive virtual reality [27].

### 4.2. Organizational Level Strategy

For the organizational level, emotional management is a variety of emotional management work based on the core of people-oriented management. Emotion management is not to suppress emotions but to allow employees to face up to their emotional state and take reasonable measures to adjust their state and give full play to their own strengths to realize human value. It should be emphasized that emotional management is inseparable from the correct counseling, which is also the main method to prevent the deterioration of employees' emotions.

As a manager, you should take the initiative to pay attention to the emotional needs of employees, provide some support when necessary, and use a more professional and systematic theoretical system to adjust the emotional state of employees from an organizational perspective. No matter how perfect the management mechanism and organizational structure are, there may be problems with the emotions of its internal employees, so it is necessary to build an emotional management system [28–30]. In terms of educational means, it is necessary to carry out various trainings and lectures to increase employees' awareness of emotional management; in terms of scientific assessment, employees can be tested by authoritative institutions to grasp the true state of employees' emotions [31, 32]. It should better meet the reasonable emotional needs of employees and provide them with necessary support. With the continuous improvement of the emotional management system, the emotional problems of employees will be better managed and controlled [33].

Organization managers need to unblock emotional problem intervention channels for employees, such as asking for emotional counseling intervention organizations to help them properly channel their negative emotions [34–36]. Some units have established their own EAP (Employee Assistance Program) specifically to address this issue, through which they can help employees manage their emotions. In fact, such an employee assistance plan is also an important manifestation of the organization's humanized management, and it is also one of the effective ways to improve the relationship between managers and employees [37]. After dealing with these problems, the efficiency of team collaboration within the organization will also be greatly improved [38].

### 4.3. Group-Level Strategies

Formal groups are interpersonal functioning groups that are formed by organizational plans and that arise within a specific workplace. Formal groups have clear organizational structures, unified goals and tasks, established disciplinary systems, fixed roles and responsibilities among members, and clear rights and obligations. Unit departments and departments belong to formal groups. The middle-level cadres and department leaders of the unit must be good at understanding the intentions of the organization and managers, treat each group member fairly, and implement humane management while strictly implementing work discipline [39, 40]. At the same time, it is necessary to understand the strengths and temperaments of employees in the department and try to mobilize the enthusiasm of subordinates, help them resolve negative emotions, and enhance collective cohesion [41]. Employees in a formal group must consciously abide by the rules and regulations of the group and actively cooperate with the implementation of the decisions made by the leaders of their departments [42].

Informal groups do not have clear organizational associations and have no established goals, tasks, and division of labor. The establishment of a group has a strong personal emotional color and is generally based on the closeness and distance between people. Therefore, informal groups are often regarded as the core of interpersonal relationships.

In informal group members, there is often a certain type of representative person who plays a central role in leading the group. This figure may be just an ordinary member of the entire organization, but he is at the center of the entire network of relationships, with unparalleled influence and appeal.

Organizational leaders can use the charisma of the core figures in the informal group to do a good job of emotional management of this group.

### 4.4. Individual-Level Strategies

Usually, the emotions of others or oneself can be judged more accurately through the physical and mental state, and only after knowing the true state of emotions can they be managed more effectively [25, 43]. It is worth noting that for emotions, there is no praise or criticism in itself. Individuals must feel and accept emotions with a real and objective state of mind. There is no doubt that only on the basis of a correct understanding of one's own emotions can one better grasp one's own emotions and show a better living and working state [44, 45].

Individuals must understand the organization's emotional management measures from the overall perspective, not engage in “small group” confrontation, not stir up personal emotions, not incite or incite colleagues around, and integrate themselves into the group. As a part of the unit, individual employees are obliged to obey the arrangement and management of the organization. Without the organization, there is no individual. Rights and obligations are complementary to each other. It is necessary to establish a healthy and progressive concept of collectivism. Only by fully cooperating with the organization's emotional management plan can we enjoy the “fruit” of emotional management.

Many employees' slackness is a matter of attitude, and some employees are unable to complete their work because of their limited business ability [46]. In addition, they neglect their studies. Over time, they form a mentality of “waiting, relying, and asking,” and they fall into boredom and procrastination [47–49]. Therefore, improving the theoretical accomplishment and improving the professional level is an effective way to change the negative attitude of employees.

## 5. Conclusion

As a new technology, virtual reality combines three-dimensional dynamic visual scenes and physical behavior systems and has the advantages of immersion, strong privacy, and design controllability. Therefore, this paper studies emotion induction from a new perspective and proposes a “virtual reality emotion induction system” to provide a more immersive and realistic way of audiovisual perception emotion induction. Through research, it is found that enterprises still need to make further improvements in the construction of corporate culture, the construction of emotional counseling system, and the clarification of human resource career planning. Since the company does not have a clear negative emotion channeling system, the expression of employees' negative emotions basically depends on their personal characteristics. Extroverted employees are more likely to express dissatisfaction, while introverted employees are more inclined to self-direction and self-solving. Therefore, the problem presents a trend of divergence between two ends. Through this research, we have reason to believe that emotional management, as an important part of the enterprise human resource management system, has a certain positive significance for the improvement of the overall business performance of the enterprise and is also an inevitable choice for the service industry to further strengthen the overall market competitiveness.

## Figures and Tables

**Figure 1:** Construction of enterprise employee emotion management system.

**Figure 2:** Statistics of people with different ratings of cultural atmosphere.

**Figure 3:** Statistics of people with different ratings of interpersonal relationships.

**Figure 4:** Weight of work happiness.

**Figure 5:** Frequency of adverse emotions before and after virtual reality technology emotional intervention.

**Table 1:** Target emotion localization.

Emotion type	Joy	Disgust	Fear	Grief	Calm
Pleasure (valence)/Std (Var)	8.15 (1.63)	3.11 (1.25)	2.89 (1.03)	2.11 (1.55)	7.07 (1.61)
Arousal (arousal)/Std (Var)	7.13 (1.19)	5.12 (1.36)	7.81 (1.42)	3.86 (1.46)	4.42 (1.24)

**Table 2:** List of multidimensional emotional features.

Feature dimension	Emotional characteristics		
Sound	Theme	Audio	Melody
Dynamic	Path phase	Moving speed	Lens conversion rate
Color	Hue	Saturation	Brightness
Intention	Prospect intention	Background intent	Environmental intention

**Table 3:** Survey results of demographic characteristics.

Basic information	Classification	Proportion (%)
Working years in this company	Within 5 years	52.3
	5-10 years	21.4
	10-15 years	14.7
	15+ years	11.6
Education	PhD	1.2
	Master	23.8
	Undergraduate	74.6
	College	2.4
Age	After 90	6.8
	After 80	50.6
	After 70	32.5
	After 60	10.1
Gender	Male	73.4
	Female	26.6

**Table 4:** Question setting and evaluation of human resource management and development.

Question	Your career development direction and career plan in the enterprise are clear	You are satisfied with the enterprise performance incentive system	Human resource department regularly conducts emotional management training and lectures
Very much in line	322	484	591
Somewhat in line	980	111	270
Not clear	341	880	23
Not quite	120	341	610
Totally inconsistent	443	390	722

**Table 5:** Question setting and evaluation of publicity and counseling.

Question	You understand emotion management	Businesses often organize activities related to emotion management	Your dissatisfaction can be communicated in a timely manner within the enterprise
Very much in line	370	291	250
Somewhat in line	484	710	570
Not clear	660	320	436
Not quite	310	203	300
Totally inconsistent	602	682	650

## Data Availability

The data used to support the findings of this study are included within the article.
